RETRACTED

# Optimizing planting geometry for barley-Egyptian clover intercropping system in semi-arid sub-tropical climate

**DOI:** 10.1371/journal.pone.0233171

**Published:** 2020-05-14

**Authors:** Muhammad Ikram ul Haq, Muhammad Mudassar Maqbool, Ansar Ali, Shahid Farooq, Shahbaz Khan, Muhammad Sohail Saddiq, Khurshied Ahmad Khan, Shahbaz Ali, Muhammad Ifnan Khan, Ansar Hussain, Muhammad Arif, Maqbool Ahmad, Mahwish Tanveer

**Affiliations:** 1 Department of Agronomy, Faculty of Agricultural Sciences, Ghazi University, Dera Ghazi Khan, Pakistan; 2 Department of Plant Protection, Harran University, Şanlıurfa, Turkey; 3 Department of Agricultural Engineering and Technology, Faculty of Agricultural Sciences, Ghazi University, Dera Ghazi Khan, Pakistan; 4 Department of Plant Protection, Faculty of Agricultural Sciences, Ghazi University, Dera Ghazi Khan, Pakistan; 5 Department of Plant Breeding and Genetics, Faculty of Agricultural Sciences, Ghazi University, Dera Ghazi Khan, Pakistan; 6 Department of Chemistry, Ghazi University, Dera Ghazi Khan, Pakistan; 7 National Institute of Food Science and Technology, Faculty of Food, Nutrition and Home Sciences, University of Agriculture, Faisalabad, Pakistan; Omer Halisdemir Universitesi, TURKEY

## Abstract

Intercropping legumes with cereals has been a common cropping system in short-season rainfed environments due to its increased productivity and sustainability. Intercropping barley (*Hordeum vulgare* L.) with Egyptian clover (*Trifolium alexandrinum* L.) could increase the grain yield of barley and improve resource use efficiency of the intercropping system. However, non-optimum planting geometry has been a hurdle in the adaptation of barley-based cropping systems. This study was aimed at optimizing the planting geometry, and assess the productivity and profitability of barley-Egyptian clover intercropping system. Ten different planting geometries, differing in number of rows of barley, width and number of irrigation furrows and planting method were tested. Intercropping barley with Egyptian clover improved 56–68% grain yield of barley compared with mono-cropped barley. Barley remained dominant crop in terms of aggressiveness, relative crowding coefficient and competitive ratio. The amount of water used was linearly increased with increasing size of barley strip from 3 to 8 rows. The highest water use efficiency (4.83 kg/cf^3^) was recorded for 8-row barley strip system with 120 cm irrigation furrows compared to rest of the planting geometries. In conclusion, 8-rows of barley planted on beds with Egyptian clover in 120 cm irrigation furrows had the highest net income and cost benefit ratio. Therefore, it is recommended that this planting geometry can be used for better economic returns of barley-Egyptian clover intercropping system. However, barley strips with >8 rows were not included in this study, which is limitation of the current study. Therefore, future studies with >8 barley rows in strip should be conducted to infer the economic feasibility and profitability of wider barley strips.

RETRACTED

## Introduction

Inefficient utilization of limited resources is one of the major constraints in crop productivity under semi-arid subtropical climates [1]. On the other hand, land area devoted to crop production has decreased due to continuous reduction in arable land in many geographic regions of the world [2, 3]. Erratic rainfall along with declining soil fertility has resulted in the failure of crops sown in monoculture. Growing low input requiring crops, water saving irrigation techniques and intercropping are the potential alternatives to maximize crop productivity and resource use efficiency [4]. Intercropping–growing of two or more crops together, which mutually benefit from the association–can mitigate the risk of crop failure [5]. If erratic rainfall affects one crop, then losses may be compensated by the additional legume crop added in the system [6]. Intercropping may provide system sustainability by allowing yield gains [7, 8]. Several problems associated with modern farming (e.g. yield stagnation, soil degradation, pest and pathogen infestation, disease incidence and environmental deterioration) could be addressed through intercropping [9]. Besides, optimum planting geometry is an important factor in different intercropping systems for better utilization of available resources and harvesting more solar radiations. Planting geometry is dependent on crop season, relative proportion of component crops, relative growth type and mechanism of yield enhancement [10].

Raised bed technology saves ~36% of water compared to conventional irrigation systems; therefore, it could improve the water use efficiency of different intercropping systems [11]. The raised bed planting system is gradually becoming popular among farmers as it allows enough light penetration [12, 13]. Several studies have reported that bed planting improved crop yield, water and nutrient use efficiencies in different crops, including crops sown in drought prone areas [12, 13].

Intercropping of legumes with cereals has been a common cropping system in short-season rainfed environments due to its increased productivity and sustainability [14]. Cereal-legume intercropping plays many roles in the agroecosystem, including improved product quality, high competitive ability against weeds and reduced negative impact of the arable crops on the environment [15]. Thus, possible advantages of raising Egyptian clover with cereals include; improved dry matter harvests, better fodder quality, less dependence on inorganic fertilization and improved succeeding crop produce [16–18]. Intercropping Egyptian clover with cereals offers the potential to partition forage yield between silage harvest and fall regrowth [19]. Intercropping Egyptian clover with barley and oat affected biomass yield, quality of fodder and composition of the species [19]. Some studies in the past have tested the effects of barley intercropped with annual fodders such as ryegrass, barseem and clover [20–22]. Biomass yield per plant of barley, oat and triticale were significantly affected by production practices, time of harvest and genotype [23]. The economics, resource use efficiency, residual soil fertility and competition among different crops sown in barley-Egyptian clover intercropping system have merely been tested in semi-arid, sub-tropical climate of Pakistan. Although, Wahla et al. [24] have studied some competitive functions of barley-based intercropping systems, a comprehensive study dealing with economics, residual soil fertility and plant geometry is missing. Therefore, the current study was conducted to test the influence of different planting geometries on productivity, profitability and residual soil fertility of barley-Egyptian clover intercropping system. It was hypothesized that intercropping will be more beneficial compared to monocropping. The results will help to optimize planting geometry for sustainable economic benefits of barley-Egyptian clover intercropping system.

RETRACTED

## Materials and methods

This study was conducted at the Agronomic Research Area, University of Agriculture, Faisalabad (latitude 31.20°N, longitude 73.06°E, 184.5 m above sea level) for two consecutive years (2014–15 and 2015–16). The region is characterized as semi-arid with very hot and humid summers and dry, cool winters. June is the hottest month with a mean maximum temperature of 40.5°C and mean minimum temperature of 26.9°C. In January, the mean minimum and maximum temperatures are 4.1°C and 19.4°C, respectively. The average annual rainfall is about 375 mm. Half of the yearly rainfall is received in July and August during the monsoon season. The weather data of both experimental years is presented in Table 1.

**Table 1:** Meteorological data during the experimental period.

		Temperature (°C)						
		Maximum	Minimum	Mean	RH (%)	Rainfall (mm)	PE (mm/24 h)	SD (h)
2014	Oct	31.3	19.1	25.2	54.6	3.6	3.5	-
	Nov	26.3	11.5	18.9	61.7	10.0	1.8	7.6
	Dec	18.5	5.9	12.2	75.0	0.0	1.5	4.7
2015	Jan	16.6	6.9	11.7	75.3	12.2	1.1	5
	Feb	22.0	11.1	16.5	66.0	20.5	2.1	5.6
	Mar	24.5	13.6	19.1	64.0	67.9	13.0	4.9
	Apr	33.2	20.7	27.0	43.9	32.8	5.3	9.1
2015	Oct	32.2	19.1	25.4	52.9	14.5	4.0	-
	Nov	27.1	12.1	19.6	61.5	8.8	2.4	6.6
	Dec	21.8	7.2	14.5	62.6	0.0	1.9	7.0
2016	Jan	17.3	7.7	12.5	74.4	13.1	3.5	1.2
	Feb	23.3	9.3	16.3	58.1	7.8	2.3	8.5
	Mar	26.8	15.6	21.2	59.7	66.7	2.7	6.6
	Apr	34.3	19.2	27.2	47.4	5.6	6.1	8.3

RH = Relative Humidity, PE = Pan Evaporation, SD = Sunshine Duration,— = no sunshine hours recorded due to clouds/fog

The soil of the experimental site was sandy clay-loam belonging Lyallpur soil series. The plough layer (20 cm) consisted of total N (0.042%), total available phosphorous (6.94 ppm) and available potassium (139 ppm) with an initial soil pH of 7.89 (Table 2). Prior to analysis, the soil samples were air-dried and sieved through a 2 mm sieve. Organic matter was determined by the Walkley and Black method. A hydrometer in a sedimentation cylinder, using sodium hexametaphosphate as the dispersing agent, was used to determine the particle size distribution. The soil reaction (pH) and electrical conductivity (EC) were measured in saturated paste.

RETRACTED

**Table 2:** Soil properties before the initiation of experiment during both experimental years.

Soil properties	2014–15	2015–16
Sand (%)	62.11	60.91
Silt (%)	18.71	17.46
Clay (%)	19.21	21.64
pH	7.89	7.81
EC (ds m^-1^)	1.15	1.12
Soil organic matter (%)	0.76	0.76
Available nitrogen (%)	0.04	0.04
Available phosphorus (ppm)	6.94	6.84
Available potassium (ppm)	139	137

*Textural class was sandy clay loam

### Experiment materials and design

Barley variety (Haider-93) and Egyptian clover variety (Anmol-2009) were used during both the experimental years. For a uniform seedbed preparation, the experimental site was ploughed three times in upper 20 cm. The experiment was laid out according to randomized complete block design with ten different planting geometries (Table 3). The size of each experimental unit was 25.2 m^2^ (3.6 m × 7.0 m), with 50 cm spacing between each unit. For various planting geometries, both crops were sown at the same time on October 10 and October 17 during 1^st^ and 2^nd^ year, respectively. Seed rate was kept 75 kg ha^-1^ and 60 kg ha^-1^ for barley and Egyptian clover, respectively. Nitrogen (N) and phosphorus (P) were applied at the rate of 50 kg ha^-1^. Half dose of N and whole P were applied at sowing, while remaining half N dose was applied with the first irrigation to barley only. A measured quantity of irrigation water was applied in furrows using a 12-inch cut-throat flume. Five irrigations were applied during the crop season. Weeds, pests and diseases were regularly controlled following integrated pest management strategies. The experiments were harvested on April 10, 2015 and April 15, 2016 during the 1^st^ and 2^nd^ year, respectively.

RETRACTED

**Table 3:** Different intercropping treatments used during both years of study.

T_1_: Barley alone sown in 30 cm spaced single rows (conventional system)
T_2_: 3-rows of barley sown on beds with 45 cm irrigation furrows
T_3_: 4-rows of barley sown on beds with 60 cm irrigation furrows
T_4_: 6-rows of barley sown on beds with 90 cm irrigation furrows
T_5_: 8-rows of barley sown on beds with 120 cm irrigation furrows
T_6_: 3-rows of barley sown on beds with Egyptian clover sown in 45 cm irrigation furrows
T_7_: 4-rows of barley sown on beds with Egyptian clover sown in 60 cm irrigation furrows
T_8_: 6-rows of barley sown on beds with Egyptian clover sown in 90 cm irrigation furrows
T_9_: 8-rows of barley sown on beds with Egyptian clover sown in 120 cm irrigation furrows
T_10_: Egyptian clover sown alone

### Data collection

All experimental units (the whole cultivated area, i.e., 25.2 m^2^) were harvested to record biological yield of both crops and grain yield of barley. The harvested units were tied into bundles and weighed for biological yield. The barley crop was manually threshed to record grain yield. The recorded biological and grain yields were converted into t ha^-1^ by unitary method. Harvest index of barley was taken as the ratio of grain to biological yield expressed in percentage. Soil samples were collected from all experimental units to assess the residual soil fertility. Prior to analysis, soil samples were air-dried, passed through 2 mm sieve and analyzed for organic matter, N, P and potassium (K) contents. Land equivalent ratio (LER), area time equivalent ratio (ATER) and barley grain yield equivalent (BGYE) were calculated to determine the advantages of different barley-Egyptian clover intercropping treatments over sole cropping [25–27]. The degree of competition and relative dominance of species within each barley-Egyptian clover intercropping treatment were assessed by calculating aggressivity (Aa), relative crowding coefficient (RCC) and competitive ratio (Cr_a_) [28–30].

The LER was calculated by following Eq 1.

$$LER=L_{ba}+L_{be}=Y_{babe}/Y_{baba}+Y_{beba}/Y_{bebe}$$ Eq 1

Here; L_ba_ = yield of intercropped barley, L_be_ = yield of intercropped Egyptian clover, Y_baba_ = pure stand yield of barley and Y_bebe_ = pure stand yield of Egyptian clover.

If LER > 1 = intercropping is advantageous over sole cropping. Similarly, if LER < 1 = intercropping is disadvantageous over sole cropping and LER = 0 means no advantage or disadvantageous of intercropping over sole cropping.

RETRACTED

The ATER was computed by following Eq 2.

$$ATER=(RY_{ba}\times t_{ba})(RY_{be}\times t_{be})/T$$ Eq 2

Here, RY_ba_ = relative yield of barley, RY_be_ = relative yield of Egyptian clover, t_ba_ = duration (days) for barley, t_be_ = duration (days) for Egyptian clover and T = duration of whole intercropping system. Relative yield was computed by dividing the biological yield in intercropping to the biological yield in sole cropping of the respective crop [31]. Grain yield equivalent of barley was calculated by converting the yield of intercrops into yield of barley based on existing market prices of each crop.

The aggressivity of barley to Egyptian clover (A_babe_) was computed by following Eq 3.

$$A_{babe}=Y_{babe}/Y_{baba}\times Z_{babe}–Y_{beba}/Y_{bebe}\times Z_{beba}$$ Eq 3

Here, A_babe_ = aggressivity of barley to Egyptian clover, Z_babe_ = sown proportion of barley in Egyptian clover and Z_beba_ = sown proportion of Egyptian clover in barley.

If A_babe_ > 0 = barley is more competitive than Egyptian clover. Similarly, if A_babe_ < 0 = Egyptian clover is more competitive than barley.

The RCC for barley (K_babe_) was computed by following Eq 4.

$$K_{babe}=Y_{babe}/Y_{baba}‐Y_{babe}\times Z_{beba}/Z_{babe}$$ Eq 4

Here, K_babe_ = RCC for barley, whereas all other abbreviations such as Y_baba_, Y_babe_, Z_babe_, Z_beba_ are described in the above equations.

The competitive ratio for barley (CR_ba_) was computed by using the Eq 5.

$$CR_{ba}=Y_{babe}/Y_{baba}\times Z_{beba}/Y_{bebe}\times Z_{beba}$$ Eq 5

Where CR_ba_ = Competitive ratio for barley and all other abbreviations such as Y_baba_, Y_babe_, Z_babe_, Z_beba_ have been described in the above equations

### Water use efficiency

Water used efficiency (WUE) of each intercropped treatment/planting geometry was calculated by dividing total dry matter produced (TDM = straw yield + grain yield) to the volume of water used (Eq 6).

WUE=TDM/volumeofwaterused Eq 6

Where TDM = total dry matter.

### Economic analysis

The data for both years were economically assessed using standard methods devised by CIMMYT [32]. These methods involve partial budgeting, marginal and sensitivity analysis. For each intercropping treatment, a partial budget was assembled to assess the expenses incurred and net returns. In the analysis, prices of inputs prevailing in the market during 2014–2015 and 2015–2016 were used to calculate the partial budget of different intercropping treatments.

### Analysis of dominance

Information delivered by the partial budget analysis did not deliver evidence in comparative gain in additional benefits from the additional costs invested in particular treatment. Therefore, analysis of dominance was executed. Treatments were organized in an ascending order from low to high cost. If the cost of the treatment stood higher and net profit was lower than foregoing treatment then such treatment was considered as "dominated" and denoted by "D".

RETRACTED

### Marginal analysis of different barley-Egyptian clover intercropping systems

In order to assess how the net field benefits from an investment on different intercropping treatments increased as the amount spent on the same increased, the marginal analysis was carried out using Eq 7.

MRR=MNF/MC×100 Eq 7

Here MRR = marginal rate of return, MNF = marginal net benefit, MC = marginal cost.

### Statistical analysis

The collected data were tested for normality by Shapiro-Wilk normality test, which indicated that some of the variables had non-normal distribution. Thus, these variables were normalized by Arcsine transformation technique. One-way analysis of variance (ANOVA) was used to test the differences between different intercropping treatments/planting geometries [33]. Least significant difference test at 5% probability was used to separate the means where ANOVA indicated significant differences [34].

## Results

### Yield and related attributes

The highest biological yield of barley (11.5 and 11.65 tons/ha in 2014–15 and 2015–16, respectively) was recorded for barley sown alone (Table 4). Among intercropping treatments, the highest biological yield (8.76, 9.05 tons/ha) was recorded for 8-rows of barley sown on beds with Egyptian clover sown in 120 cm irrigation furrows and the lowest (8.39, 8.46 tons/ha) was recorded for 3-rows of barley sown on beds with Egyptian clover cultivated in 45 cm irrigation furrows for both crop seasons.

**Table 4:** Influence of different barley-Egyptian clover intercropping techniques on biological and grain yields, and harvest index of barley.

	Biological yield (t ha^-1^)		Grain yield (t ha^-1^)		Harvest index (%)	
Treatments	2014–15	2015–16	2014–15	2015–16	2014–15	2015–16
Barley alone at 30 cm spaced single rows	11.50 A	11.63 A	3.84 A	3.92 A	33.98 A	35.22 A
3-rows of barley on beds with 45 cm irrigation furrows	11.05 AB	11.24 A	3.62 B	3.67 B	33.20 AB	33.05 B
4-rows of barley on beds with 60 cm irrigation furrows	10.57 BC	11.18 A	3.45 B	3.62 B	33.62 ABC	31.73 BC
6-rows of barley on beds with 90 cm irrigation furrows	10.51 BC	10.89 A	3.47 B	3.66 B	33.80 A	31.71 C
8-rows of barley on beds with 120 cm irrigation furrows	10.15 C	11.00 A	3.42 B	3.68 B	33.39 A	31.01 C
3-rows of barley on beds with Egyptian clover in 45 cm irrigation furrows	8.39 D	8.46 B	2.59 C	2.76 E	31.69 BCD	31.59 C
4-rows of barley on beds with Egyptian clover in 60 cm irrigation furrows	8.56 D	8.57 B	2.65 CD	2.86 D	31.15 CD	30.86 C
6-rows of barley on beds with Egyptian clover in 90 cm irrigation furrows	8.44 D	9.03 B	2.82 C	3.08 C	30.87 D	30.79 C
8-rows of barley on beds with Egyptian clover in 120 cm irrigation furrows	8.76 D	9.05 B	2.84 C	3.27 C	30.63 D	30.75 C
*LSD (p≤0*.*05)*	*0*.*72*	*1*.*09*	*0*.*21*	*0*.*32*	*1*.*51*	*1*.*32*

Means sharing the same letter within a column or a row do not differ significantly (p > 0.05).

RETRACTED

The highest grain yield of barley (3.84, 3.92 tons/ha for 2014–15 and 2015–16, respectively) was recorded for barley alone treatment (Table 4). Among intercropping treatments the highest grain yield of barley (2.84, 3.27 tons/ha for 2014–15 and 2015–16, respectively) was recorded for 8-rows of barley sown on beds with Egyptian clover sown in 120 cm irrigation furrows. Three rows of barley sown on beds with Egyptian clover cultivated in 45 cm irrigation furrows had the lowest grain yield (2.58, 2.76 tones/ha) for both crop years.

Harvest index varied across different barley-Egyptian clover intercropping treatments (Table 4). The highest harvest index was recorded for barley cultivated alone in 30 cm rows followed by 6-rows of barley sown on beds with 90 cm irrigation furrows during 2014–15. Different trend was observed during 2015–16 where the highest harvest index (35.22%) was noted for barley sown alone in 30 cm rows followed by 3-rows of barley cultivated on beds with 45 cm irrigation furrows. The lowest harvest index (30.6%, 30.8% in 2014–15 and 2015–16, respectively) was recorded for 8-rows of barley sown on beds with Egyptian clover cultivated in 120 cm irrigation furrows (Table 4).

The highest fodder yield of Egyptian clover (68.33, 69.83 tons/ha) for both years was recorded for Egyptian clover cultivated alone (Table 5). Among intercropping treatments, the highest fodder yield (56.67, 58.67 tons/ha during 2014–15 and 2015–16, respectively) was recorded for 8-rows of barley sown on beds with Egyptian clover cultivated in 120 cm irrigation furrows. The lowest fodder yield (21.33, 21.00 tons/ha during 2014–15 and 2015–16, respectively) was recorded for 3-rows of barley cultivated on beds with Egyptian clover sown in 45 cm irrigation furrows (Table 5).

**Table 5:** Fodder yield of Egyptian clover as influenced by different barley-Egyptian clover intercropping treatments.

	Fodder yield (t ha^-1^)	
Treatments	2014–15	2015–16
3-rows of barley on beds with Egyptian clover in 45 cm irrigation furrows	21.33 C	21.00 E
4-rows of barley on beds with Egyptian clover in 60 cm irrigation furrows	25.67 C	29.33 D
6-rows of barley on beds with Egyptian clover in 90 cm irrigation furrows	31.67 C	35.12 C
8-rows of barley on beds with Egyptian clover in 120 cm irrigation furrows	56.67 B	58.67 B
Egyptian clover alone	68.33 A	69.83 A
*LSD (p≤0*.*05)*	*1*.*68*	*2*.*13*

Means sharing the same letter within a column or a row do not differ significantly (p > 0.05). Treatments lacking barley were omitted

RETRACTED

### Aggressivity/Competitive ratio/relative crowding coefficient

The highest value of aggressivity (+0.65) was noted for 6-rows of barley sown on beds with Egyptian clover cultivated in 90 cm irrigation furrows during 2014–15. During the second year, barley was more competitive in 3-rows of barley sown on beds with Egyptian clover cultivated in 45 cm irrigation furrows compared to the rest of the intercropping treatments. In terms of relative crowding coefficient (RCC), the highest value (66.8, 79.5) was recorded for 8-rows of barley sown on beds with Egyptian clover cultivated in 120 cm irrigation furrows for both crop years, while the lowest (25.8, 30.2) was recorded for 3-rows of barley sown on beds with Egyptian clover cultivated in 45 cm irrigation furrows. The highest value of competitiveness (4.95, 4.09) for both years was recorded for 8-rows of barley cultivated on beds with Egyptian clover sown in 120 cm irrigation furrows (Table 6).

**Table 6:** Competitive functions of barley as influenced by different barley-Egyptian clover intercropping treatments.

	Aggressivity				Relative crowding coefficient						Competitive ratio			
	2014–15		2015–16		2014–15		2015–16			2014–15			2015–16	
Treatments	Barley	IC	Barley	IC	B	IC	Sys	B	IC	Sys	Barley	IC	Barley	IC
3-rows of barley on beds with Egyptian clover in 45 cm irrigation furrows	0.62	-0.62	1.07	-1.07	2.83	9.15	25.8	3.35	9.03	30.2	0.03	0.30	0.03	0.22
4-rows of barley on beds with Egyptian clover in 60 cm irrigation furrows	0.63	-0.63	0.86	-0.86	2.84	10.6	30.1	3.11	10.6	33.1	0.04	0.60	0.04	0.50
6-rows of barley on beds with Egyptian clover in 90 cm irrigation furrows	0.65	-0.65	0.74	-0.74	2.90	13.1	37.9	2.92	14.4	42.1	0.07	2.64	0.06	1.70
8-rows of barley on beds with Egyptian clover in 120 cm irrigation furrows	0.17	-0.17	0.45	-0.45	2.95	22.6	66.8	3.39	23.4	79.5	0.08	4.95	0.08	4.09

IC = Intercrop, B = Barley, Sys = System, the treatments where barley had no competition with Egyptian clover were omitted

### LER/ATER/BGYE

In the first year, the values of LER were >1.00 in all intercropping treatments showing a yield advantage of intercropping over monocropping (Table 7). The highest value of LER (1.56) was recorded for 8-rows of barley sown on beds with Egyptian clover cultivated in 120 cm irrigation furrows. In the second year, LER in all intercropping treatments was >1.00 with the highest value (1.68) recorded for 8-rows of barley sown on beds with Egyptian clover cultivated in 120 cm irrigation furrows. There was a similar trend for ATER, but values were lower than LER. The highest value of ATER (1.54, 1.61 during 2014–15, 2015–16, respectively) was recorded for 8-rows of barley sown on beds with Egyptian clover cultivated in 120 cm irrigation furrows. All intercropping treatments showed a yield advantage over monocropping during both years. The 8-rows of barley cultivated on beds with Egyptian clover sown in 120 cm irrigation furrows was a superior treatment with the highest value of BGYE (125.0%, 121.1% in 2014–15 and 2015–16, respectively) (Table 7).

RETRACTED

**Table 7:** Agronomic advantages of barley as influenced by different barley-Egyptian clover intercropping treatments.

	Land equivalent ratio		Area time equivalent ratio		Barley grain yield equivalent (%)	
Treatments	2014–15	2015–16	2014–15	2015–16	2014–15	2015–16
3-rows of barley on beds with Egyptian clover in 45 cm irrigation furrows	1.06	1.10	1.02	1.08	21.67	8.67
4-rows of barley on beds with Egyptian clover in 60 cm irrigation furrows	1.03	1.11	1.03	1.04	33.51	27.45
6-rows of barley on beds with Egyptian clover in 90 cm irrigation furrows	1.16	1.19	1.11	1.12	59.01	47.07
8-rows of barley on beds with Egyptian clover in 120 cm irrigation furrows	1.56	1.68	1.54	1.61	124.96	121.09

Treatments where barley had no competition with Egyptian clover were omitted

### Water use efficiency

Different planting geometries significantly influenced water use efficiency (WUE) (Table 8). The highest WUE (4.8 kg cf^3^) was recorded for 8-rows of barley sown on beds with Egyptian clover intercropped in 120 cm irrigation furrows and the lowest (1.49 cf^3^) WUE was recorded for barley cultivated alone in 30 cm rows. Amount of water saved in different treatments ranged between 15.1–28.3%. Additional area that can be irrigated from this saved water for raising sole barley ranged between (0.15–0.28 ha). Additional yield of barley that can be achieved with the saved amount of water ranged between 1.75–3.27 tons/ha (Table 8).

**Table 8:** Water related attributes as influenced by different barley-Egyptian clover intercropping treatments.

Treatments	Total water applied (cubic ft. per ha)	Irrigation water use efficiency kg cf^3^	Percent saving water (cubic ft. per ha)	Additional area (ha) that can be brought under cultivation by saved irrigation water	Additional yield of barley (t ha^-1^) that can be obtained by saved irrigation water
Barley alone at 30 cm spaced single rows (conventional system)	776182	1.49	-	-	-
3-rows of barley on beds with 45 cm irrigation furrows	567454	1.96	26.6	0.27	3.07
4-rows of barley on beds with 60 cm irrigation furrows	580269	1.87	24.9	0.25	2.88
6-rows of barley on beds with 90 cm irrigation furrows	554097	1.93	28.3	0.28	3.27
8-rows of barley on beds with 120 cm irrigation furrows	619435	1.71	19.9	0.20	2.30
3-rows of barley on beds with Egyptian clover in 45 cm irrigation furrows	564358	2.98	27.0	0.27	3.11
4-rows of barley on beds with Egyptian clover in 60 cm irrigation furrows	589313	3.15	23.8	0.24	2.75
6-rows of barley on beds with Egyptian clover in 90 cm irrigation furrows	578905	3.83	25.1	0.25	2.90
8-rows of lentil on beds with Egyptian clover in 120 cm irrigation furrows	654924	4.83	15.1	0.15	1.75
Egyptian clover alone	1069877	2.56	-39.1	-0.39	-4.51

RETRACTED

### Residual soil fertility in different barley-Egyptian clover intercropping systems

Postharvest soil analysis revealed that all intercropping treatments had higher percentage of organic matter compared to sole treatments (Table 9). Organic matter was significantly higher in treatments where Egyptian clover was intercropped with barley. The highest organic matter percentage (0.67, 0.68%) was recorded for 8-rows of barley sown on beds with Egyptian clover intercropped in 120 cm irrigation furrows followed by 6-rows of barley cultivated on beds with Egyptian clover sown in 90 cm irrigation furrows (0.59, 0.61%) during 2014–15 and 2015–16, respectively. The N percentage also varied among treatments during both years. Egyptian clover showed a positive effect on N percentage. The highest N percentage (0.041, 0.043%) was recorded for Egyptian clover cultivated alone followed by 8-rows of barley sown on beds with Egyptian clover intercropped in 120 cm irrigation furrows for both crop years (Table 9).

**Table 9:** Residual soil fertility as influenced by different barley-Egyptian clover intercropping treatments.

	Organic matter (%)		Nitrogen (%)		Phosphorus (%)		Potassium (ppm)	
Treatments	2014–15	2015–16	2014–15	2015–16	2014–15	2015–16	2014–15	2015–16
Barley alone at 30 cm spaced single rows	0.48	0.43	0.025	0.027	8.25	8.45	246	241
3-rows of barley on beds with 45 cm irrigation furrows	0.47	0.45	0.031	0.030	6.25	6.77	235	230
4-rows of barley on beds with 60 cm irrigation furrows	0.48	0.47	0.035	0.032	7.63	7.63	231	233
6-rows of barley on beds with 90 cm irrigation furrows	0.49	0.46	0.030	0.034	6.14	6.68	236	234
8-rows of barley on beds with 120 cm irrigation furrows	0.45	0.48	0.032	0.035	7.85	7.68	237	233
3-rows of barley on beds with Egyptian clover in 45 cm irrigation furrows	0.50	0.49	0.036	0.038	5.81	5.60	225	226
4-rows of barley on beds with Egyptian clover in 60 cm irrigation furrows	0.56	0.59	0.037	0.039	6.27	6.56	229	227
6-rows of barley on beds with Egyptian clover in 90 cm irrigation furrows	0.59	0.61	0.038	0.040	6.50	7.65	244	233
8-rows of barley on beds with Egyptian clover in 120 cm irrigation furrows	0.67	0.68	0.040	0.041	6.40	5.71	231	234
Egyptian clover alone	0.53	0.55	0.041	0.043	6.39	5.68	235	225

RETRACTED

### Economic analysis

The highest net income (1749.58 US$) was obtained against the total cost of (1142.57 US$) in 8-rows of barley sown on beds with Egyptian clover cultivated in 120 cm irrigation furrows with the highest value (2.53) of benefit: cost ratio (BCR). The lowest net return (653.90 US$) was noted for 8-rows of barley on beds with 120 cm irrigation furrows against the total cost of (1043.91 US$) with 1.63 BCR (Table 10).

**Table 10:** Economic analysis as influenced by different barley-Egyptian clover intercropping treatments.

Treatments	Gross benefit (US$ ha^-1^)	Variable cost (US$ ha^-1^)	Fixed cost (US$) ha^-1^)	Total cost (US$ ha^-1^)	Net income (US$ ha^-1^)	BCR
barley alone at 30 cm spaced single rows (conventional system)	1858.60	222.64	848.39	1071.03	787.57	1.74
3-rows of barley on beds with 45 cm irrigation furrows	1759.20	213.59	848.39	1061.98	697.22	1.66
4-rows of barley on beds with 60 cm irrigation furrows	1709.80	202.14	848.39	1050.53	659.27	1.63
6-rows of barley on beds with 90 cm irrigation furrows	1716.80	200.14	848.39	1048.53	668.27	1.64
8-rows of barley on beds with 120 cm irrigation furrows	1697.80	195.52	848.39	1043.91	653.90	1.63
3-rows of barley on beds with Egyptian clover in 45 cm irrigation furrows	1846.12	249.49	848.39	1097.88	748.24	1.68
4-rows of barley on beds with Egyptian clover in 60 cm irrigation furrows	2036.10	270.25	848.39	1098.65	937.46	1.85
6-rows of barley on beds with Egyptian clover in 90 cm irrigation furrows	2249.87	285.41	848.39	1103.80	1146.08	2.04
8-rows of barley on beds with Egyptian clover in 120 cm irrigation furrows	2892.15	294.18	848.39	1142.57	1749.58	2.53
Egyptian clover alone	1727.00	123.02	848.39	971.41	878.61	2.04

BCR = benefit:cost ratio

### Dominance/marginal analysis

The 4-rows of barley sown on beds with 60 cm irrigation furrows, followed by 8-rows of barley cultivated on beds with 120 cm irrigation furrows and 3-rows of barley sown on beds with Egyptian clover intercropped in 45 cm irrigation furrows were dominant treatments. The dominated treatments were less productive and profitable than raising barley as sole crop. The highest marginal rate of return (6882%) was attained from 8-rows of barley sown on beds with Egyptian clover cultivated in 120 cm irrigation furrows (Table 11).

**Table 11:** Dominance/ marginal analysis of different barley-Egyptian clover intercropping treatments.

Treatments	Variable cost (US $)	Net income (US $)	Dominance	Marginal cost (US $)	Marginal net benefit (US $)	MRR%
Egyptian clover alone	12302	75157	-	-	-	-
8-rows of barley on beds with 120 cm irrigation furrows	19551	64864	D	-	-	-
6-rows of barley on beds with 90 cm irrigation furrows	20014	66827		463	1963	424
4-rows of barley on beds with 60 cm irrigation furrows	20214	65649	D	-	-	-
3-rows of barley on beds with 45 cm irrigation furrows	21359	69444		1145	3795	331
Barley alone at 30 cm spaced single rows	22264	78479		905	9035	998
3-rows of barley on beds with Egyptian clover in 45 cm irrigation furrows	24949	74143	D	-	-	-
4-rows of barley on beds with Egyptian clover in 60 cm irrigation furrows	27025	93064		2076	18921	912
6-rows of barley on beds with Egyptian clover in 90 cm irrigation furrows	28541	113925		1516	20861	1376
8-rows of barley on beds with Egyptian clover in 120 cm irrigation furrows	29418	174277		877	60351	6882

D = Dominated treatments,— = dominated treatments were lacking in MRR analysis, MRR = marginal rate of return

RETRACTED

## Discussion

Barley and Egyptian clover raised as sole crops produced significantly higher biological and grain yields compared to barley-Egyptian clover intercropping treatments during both years. The final yield of a crop is a collective effect of agronomic, genetic and environmental conditions [35]. Barley and Egyptian clover yields were reduced by intercropping and planting geometries established with different planting intensities [24]. The competition within both companion crops might be a reason of yield declined. This is a clear indication that functional ability of barley to convert dry matter into biological/grain yield is significantly affected by various intercropping treatments. Harvest index also differed among different barley-Egyptian clover intercropping treatments. This could be explained by variable competition among plants due to different planting intensities within each intercropping treatment. Harvest index was higher during the second year compared to the first year due to more ideal environmental conditions. Both sole crops produced higher yields with efficient utilization of applied inputs due to a competition-free environment compared to intercropping. Numerous studies conducted in the past have reported that intercropping decreased crop yield compared to sole sown crops [15, 36]. The degree of competition was quite variable for both crops. Barley was more competitive and a dominant crop than Egyptian clover throughout the study. Barley utilized resources (e.g. light, water and nutrients) more efficiently than Egyptian clover. Egyptian clover is a short statured crop and its low competitive ability could be attributed to the shading effect of barley. Land equivalent ratio and barley grain yield equivalent are important to determine the advantages of intercropping over sole cropping systems. The values of LER and BGYE were higher during the second year compared to the first year. The differences in LER and BGYE values might be due to more favorable growth conditions during the second year compared to the first year. Similar findings were also reported by Mandal et al. [37] in wheat + chickpea and wheat + brassica intercropping systems. Similarly, Rai [38] found that LER of all legume intercrops showed a yield advantage in case of buffel grass intercropped with annual grain legume crops.

RETRACTED

Bed planting caused substantial saving of irrigation water over traditional irrigation systems. This water saving might be attributed to the reason that in all intercropped treatments, a measured quantity of irrigation water was applied only to irrigation furrows keeping in view the water requirement of the crop sown. The crop sown on upper beds gets water through seepage. There was progressive increase in the amount of water saved and yield with increasing bed and irrigation furrow size over conventional the flat irrigation system. The water saving is directly related with the increasing bed size, which decreased the amount of irrigation water applied in the furrows. However, larger bed size (i.e., >8 barley rows) was not included in current study which should be regarded as limitation of the study. Irrigation water saving was 36–40% on wide beds, 34–31% on medium beds and 7–8% on narrow beds, for wheat and maize crops respectively, when compared with flood irrigation. Cereal-legume intercropping improves soil structure due to legume intercrop by aggregation around root hairs by fine soil particles [39], with economic use of capital and labor [40]. In the current study, organic matter and nitrogen increased, while phosphorus and potassium were decreased in the treatments where Egyptian clover was intercropped with barley. The reason of high organic matter and nitrogen percentage was due to Egyptian clover (legume crop) which added nitrogen into soil through biological nitrogen fixation. The profitability and feasibility of an intercropping system is reflected through economic returns [41, 42]. Barley-Egyptian clover intercropping was economically more profitable than sole cropping in terms of net benefit with low cost of production. Cost of production was higher with low benefit:cost ratio in sole sown crops compared to intercropping treatments.

Barley intercropped with Egyptian clover on raised beds along with precise application of water used resources more efficiently than sole crop stands. The losses caused by intercropping were compensated by the component crops. In another study, the highest net returns were obtained when sorghum was intercropped with groundnut, soybean and pigeon pea with 3:3 row ratios compared to sole crops [43]. Similarly, intercropping of sorghum and soybean in different row arrangements gave the highest net returns compared to the sole crops [44]. Significantly higher net field benefits of different intercropping systems in cotton, rice and wheat has also been reported by Khan [45].

RETRACTED

## Conclusion

Intercropping 8-rows of barley sown on beds with Egyptian clover cultivated in 120 cm irrigation furrows performed better and appeared as most promising treatment in terms of sustainability, profitability and irrigation water use efficiency. This intercropping treatment could be used to improve the productivity and profitability of barley-Egyptian clover intercropping system in semi-arid, sub-tropical climates. However, barley strips with >8 rows were not included in this study, which is limitation of the current study. Therefore, future studies with >8 barley rows in strip should be conducted to infer the economic feasibility and profitability of wider barley strips.
